# Efficacy and Safety of Remimazolam Besylate Combined with Alfentanil in Painless Gastroscopy: A Randomized, Single-Blind, Parallel Controlled Study

**DOI:** 10.1155/2022/7102293

**Published:** 2022-09-22

**Authors:** Chang Xu, Long He, Juanjuan Ren, Junfei Zhou, Haiming Guo, Na Chen, Hongfei Chen, Yunqi Lv

**Affiliations:** Department of Anesthesiology, Pain and Perioperative Medicine, The First Affiliated Hospital of Zhengzhou University, Zhengzhou 450052, China

## Abstract

**Background:**

The efficacy and adverse reactions of remimazolam besylate (RB) in combination with alfentanil in patients with painless gastroscopy remain unclear.

**Objective:**

The aim of the study is to observe the efficacy and adverse reactions of RB in combination with alfentanil in patients with painless gastroscopy RB.

**Methods:**

All patients were randomly divided into two groups: RB combined with the alfentanil group (research group) and propofol combined with the alfentanil group (control group). After full oxygen inhalation and electrocardiographic monitoring, the research group was given 10 *μ*g/Kg alfentanil + RB 0.2 mg/kg intravenously, and the control group was given 10 *μ*g/Kg alfentanil + propofol 1.5 mg/kg. If there is a clinical need, the research group was given 2.5 mg/additional RB, whereas the control group was treated with an additional 0.5 mg/kg propofol. Main outcome measures were as follows: The vital endpoints including diachronic changes in heart rate (HR), blood pressure (BP), respiratory rate (RR), blood oxygen saturation (SPO_2_), end-expiratory carbon dioxide (etCO_2_), IPI, modified observer's assessment of alert/sedation (MOAA/S), time-related endpoints, perioperative adverse events, endoscopy, and anesthesiologist satisfaction, and 24-hour follow-up of adverse reactions, IPI scores, and satisfaction were recorded.

**Results:**

The HR and BP of the patients in the research group and the control group decreased, with a greater decrease in the control group, and the difference was statistically significant (*p* < 0.05). The values of RR, PETCO_2_, and IPI in the research group and the control group decreased to the lowest at 2–3 min but the decrease in the control group was more significant. Furthermore, there was no significant difference in the time from the completion of administration to 4 minutes of IPI and the total examination time, but the awakening time in the research group was slightly longer than that in the control group, and the difference was statistically significant (*p* < 0.05). The incidences of respiratory depression and hypotension during the operation were shown to be markedly smaller in the investigation relative to the control team, and the difference was statistically significant (*p* < 0.05), whereas the occurrence of cough, movements, and singultus was more common in the investigations, and the difference was statistically significant (*p* < 0.05). The results of the 24-hour follow-up showed that the adverse reactions such as nausea, dizziness, fatigue, abdominal pain, and abdominal distension were much less frequent in the study team, and the difference was statistically significant (*p* < 0.05), and the patient satisfaction was higher than in the control group, and the difference was statistically significant (*p* < 0.05). The regression results showed that age, sedative, and total dose of analgesia had significant effects on the results, and the covariance coefficient of sedative was 1.57 of IPI score in the research group higher than that of the control group.

**Conclusions:**

RB combined with alfentanil can provide safe and effective sedation for patients undergoing painless gastroscopy. Compared with propofol, RB and alfentanil for injection can avoid large hemodynamic fluctuations and deep sedation, and have fewer adverse reactions. However, the cases involved in this study are all from a single-center data, which requires further multicenter research and conformation.

## 1. Introduction

Painless gastroscopy is defined as gastroscopy on patients under sedation, which serves an essential part in the diagnostic and therapeutic approach of digestive problems, owing to its advantages such as safety, short operation time, high diagnosis rate, and good adaptability of patients [1]. In view of the environmental pollution of the operating room, the application of intravenous anesthetics is significantly higher than that of inhaled anesthetics [2]. At present, the main drugs commonly used in painless gastroscopy [3] are propofol, etomidate, midazolam, fentanyl, sufentanil, remifentanil, and dexmedetomidine.

At the beginning of the 21st century, the continuous emergence of new drugs led to the rapid development of intravenous anesthesia. Remimazolam besylate (RB) is an ultra-short-acting benzodiazepine drug that acts on GABA receptors to induce sedation [6]. Thus, RB could be developed for sedation during therapeutic and diagnostic operations, induction, and maintenance of anesthesia [6]. The pharmacokinetics of remimazolam were linear, with clearance not linked to body weight, and long-term or high-dose intravenous infusion would not cause drug accumulation. Through the evaluation of pharmacokinetics and pharmacodynamics, compared with midazolam, the change in volume-dependent half-life with infusion time is very small and is not affected by infusion time. At present, remimazolam has been under phase III clinical studies in many fields, such as colonoscopy, fiberoptic bronchoscopy, induction, and maintenance of anesthesia [7–10]. The effect of remimazolam in anesthesia is not inferior to propofol, with fewer hemodynamic side effects, and can play an important role in preventing intraoperative hypotension as a new choice of moderate sedatives [9].

Alfentanil conducted for patients undergoing daytime surgery has many advantages, such as quick effect, fast recovery, high safety, and good analgesic effect, which could retain autonomous breathing, not easily induce cough, low incidence of PONV, less pain sensitivity [11, 12]. One important reason was the inhibition of the cardiovascular system by fentanyl analgesics such as propofol and remimazolam, which is related to their pharmacological properties. However, there is a greater decrease in the propofol combined with the alfentanil group, which indicates that RB has a less cardiovascular effect than propofol, and the changes of HR, BP are relatively stable, which is also consistent with the conclusions of previous drug clinical trials [13].

In this randomized, single-blind, parallel controlled study, patients undergoing painless gastroscopy were given intravenous anesthesia with alfentanil combined with RB to observe the effects on hypertension, heart rate, oxygen saturation, muscle tremor, injection soreness, and other intraoperative and postoperative adverse reactions, and to explore the safety and comfort of alfentanil combined with RB in patients undergoing painless gastroscopy.

## 2. Methods

### 2.1. Ethical Statement

This study is a randomized controlled study. The Ethics Board for Science and Technology and Preclinical at Zhengzhou University's first medical university approved the study (Chairperson, Professor Li Tian) on 20 July 2020 (2020-KY-421), and it was performed from January 2021 to March 2021. This trial is already enrolled in the National Registry of Medical Research in China (Registry No.：ChiCTR2000040058). All the supporting documents can be found in the supplementary materials. General clinical data in the research group and control group are shown in Figure 1 and Table 1.

### 2.2. Case Selection

#### 2.2.1. Selection Criteria

This study was conducted in the 1st affiliated hospital of Zhengzhou University's Department of Anesthesiology, Pain, and Perioperative Medicine. Patients according to the order of entering the group, and then the statistician according to the randomization method to use professional statistical software to generate a random number (The block-rand software R4.0.2 [R Foundation for Statistical Computing, Vienna, Austria] generates cluster randomized numbers.) to enter the research group or the control group, in turn, do not skip or choose drugs independently. After determining the group of patients, the medicine was given according to the plan by two of the same anesthesiologists. If any of the following items is “No”, the subjects are not allowed to participate in the trial: (1) patients with gastroscopy without sedation; (2) 18–85 years old, regardless of gender; (3) the American Association of Anesthesiologists is classified as Grade -III by the American Association of Anesthesiologists.

#### 2.2.2. Exclusion Criteria

If any of the following is “yes”, the subjects are not allowed to participate in the trial: (1) patients undergoing emergency surgery; (2) patients who need endotracheal intubation for general anesthesia; and (3) cases with incomplete data.

#### 2.2.3. Elimination Standard

The study should be excluded if the following occurs: (1) patients who withdraw their informed consent without giving reasons for the decision; (2) patients who do not meet the enrollment criteria or exclusion criteria; and (3) loss of follow-up.

### 2.3. Research Program

According to the randomized grouping table, the treatment regimen was divided into two groups: alfentanil combined with RB group: The recommended regimen was 10 *μ*g/kg + remimazolam 0.2 mg/kg, and remimazolam could be added at 2.5 mg/times according to the condition of the patients during the operation. Alfentanil combined with propofol group: the recommended regimen was 10 *μ*g/kg + propofol 1.5 mg/kg. Propofol 0.5 mg/kg can be added during the operation according to the condition of the patient.

Hypotension was defined as a drop in SBP of less than 90 mmHg. The study used Ephedrine 3–5 mg to deal with aortic hypotension, described as an SBP of 80 mm Hg or a reduction of over 30% versus pretherapy SBP. Bradycardia was determined as a drop in HR to 60 beats/min; in the event of a reduction in HR to <50 beats/min, an intravenous dose of atropine 0.3–0.5 mg was prescribed. All patients fasted for at least 8 hours and water for at least 2 hours before the operation. After entering the room, the venous passage was established in the right arm with a 24 g indwelling needle. The nasal catheter of the Capno bedside monitor inhaled oxygen (oxygen flow rate of 4-5 L/min). Blood pressure, heart rate, SPO_2_, PetCO_2,_ and IPI were monitored routinely. The left arm is used to measure blood pressure, spare anesthetic machines, simple respirators, and rescue medicine, etc.

### 2.4. Observing Items and Testing Time Points

#### 2.4.1. General Indicators

Age, sex, BMI, ASA grade, past history (including history of PONV or motion sickness), and time of fasting before operation are general indicators. The amount of fluid replacement, preinhalation of oxygen, and the flow rate of inhaled oxygen were recorded. Apfel score of patients: female, nonsmoking, experience of PONV or movement illness, and postoperatively opioid usage were the four primary risk factors for adulthood PONV. Each component was given a score of 0, 1, 2, 2, 3, 4.

#### 2.4.2. Main Evaluation Endpoints

The lowest value of the integrated pulmonary index (IPI). The IPI index is considered a new indicator approved by the FDA to reflect the respiratory state of patients during sedation [14]. IPI is a comprehensive index on the basis of four specific biological variables: end-expiratory carbon dioxide (etCO_2_), respiratory rate (RR), blood oxygen saturation (SPO_2_), and pulse rate (PR). IPI values range from 1 to 10, of which 10 represents the best lung state.

#### 2.4.3. Secondary Evaluation Endpoints

1. Including blood pressure, heart rate, SPO_2_, respiratory rate, and MOAAS sedation depth score. Monitoring time: 1–3 before induction, 1 min, 3 min, 6 min, 9 min, 12 min, 15 min, 20 min after induction, and at the end of the operation. MOAA/S score: 5 score: normal tone calls the subject's name to respond quickly. 4 score: the normal tone calls for the subjects' names to be slow to respond. 3 score: call the subject's name loudly and/or repeatedly before there are response. 2 score: respond to slight acupuncture or shaking. 1 score: reaction to a strong compression of trapezius muscle; 0 score: no response to a strong compression of the trapezius muscle.
2. *Time-related endpoints*
3. Effective time: The time from administration to effect on patients.
4. The time interval from the completion of drug administration to the time when IPI reaches 4 points.
5. Total examination time (the time it takes from the beginning of the endoscopy to the exit of the endoscope). If the inspection is temporarily interrupted due to a sedation-related adverse event, the time is subtracted from the total examination time.
6. Awakening time (recording the time from drug withdrawal to the time the patient opens his eyes).
7. *The type and dose of drugs used during operation*.
8. The total dose of propofol or RB.
9. *Other adverse events during the operation*:
10. Hypotension, airway obstruction, respiratory depression, apnea, bradycardia, tachycardia, intraoperative awareness, body movement, etc.
11. Patient satisfaction, anesthesiologist satisfaction, and endoscopic physician satisfaction (VAS score)

Before patients left PACU, endoscopic physician satisfaction and anesthesiologist satisfaction were evaluated. During the telephone follow-up 24 hours after the operation, the satisfaction of the patients was evaluated, and whether the patients were willing to undergo endoscopy or not was recorded. The satisfaction score was scored by the VAS method, with a long 10 cm swimming scale with 10 scales, with 0 and 10 points at both ends, respectively. The patients were asked to mark the corresponding position on the ruler that could represent their comfort degree, and the observes scored them according to the position marked by the patients. A mark of 0 indicates utmost displeasure, whereas a mark of 10 indicates complete pleasure. (6) Adverse reactions 24 hours after operation.

24 hours after operation, the adverse reactions were divided into mild, moderate and severe grades according to nausea, vomiting, dizziness, abdominal distension, and somnolence. The frequency of vomiting within 24 hours after the operation was recorded.

### 2.5. Statistical Analysis

The average IPI score in 3 min was used as an evaluation index for sample size estimation. In our study, we selected 140 patients, including 70 patients in the research group and 70 patients in the comparison cohort. The average IPI score of the research group was 5.370 ± 1.403, and the average IPI score of the control group was 5.116 ± 1.168. Suppose X ∼ N (5.370, 1.967), Y ∼ N (5.116,1.364), the test level and effectiveness are the ratio of the sample size of the test group to the control group. We use the following formula to calculate the sample size of two groups of samples, where *zα*1/2 and *z*_*β*_ are the alpha and beta risks and *d* is Cohen's d: (*m*_1_ − *m*_2_)/SD.

(1) $$\begin{array}{c} n={\left[\frac{\left(z_{\alpha /2}+z_{\beta }\right)}{d}\right]}^{2}. \end{array}$$

A SQLite database was applied for data management; IBMSPSS24.0 software was applied for statistical analysis. The measurement data were expressed by mean ± standard deviation. The counting data were expressed by frequency or rate. The *T* test was used when measurement data obeyed normal distribution, and the rank sum test was used when it did not obey normal distribution. A *χ*^2^ test was used to compare the classified counting data. Repeated measurement data were analyzed by repeated measurement analysis of variance. Main effect test results were used when there was no interaction, and simple effect analysis was carried out when there was interaction. *p* < 0.05 indicates that the difference between groups is statistically significant.

## 3. Results

### 3.1. Comparison of General Clinical Data

In terms of gender, past history, surgical history, smoking history, alcoholism, motion sickness history, PONV, ASA grading height, weight, and age, the results showed that no large discrepancy was discovered between the controlled and research groups.

### 3.2. Comparison of Vital Signs

After administration, the blood pressure, heart rate, respiratory rate, PETCO_2_, SPO_2,_ and IPI of the patients in the research group and the control declined to varying degrees, and the difference was statistically significant (*p* < 0.05).

The systolic blood pressure in the research group was considerably greater than that control group when inserting the gastroscope, after administration, 1 min, 2 min, 3 min, 5 min, 7 min, and at the end of the operation. The diastolic BP in the research group was significantly larger than control's when complete insertions of a gastroscope, after administration, 1 min, 2 min, 3 min, 5 min, 7 min, 10 min, and at the end of the operation. The HR of the research group was higher than that of the control at 1.5 min, 2 min, 2.5 min, 3 min, 5 min, 7 min, and 10 minutes after administration, indicating that the inhibition of heart rate in the research group was mild. The value of 0.5 min in the test cohort was less than that of the control group at baseline and after administration, but at 1.5 min, 2 min, 2.5 min, 3 min, and 5 min after administration, the PETCO_2_ in the control group decreased sharply, which was lower than that in the research group. After administration of 10 min and at the end of the operation, PETCO_2_ in the control group increased again, which existed larger than of the research group, and there are statistically significant differences between groups (*p* < 0.05). The respiratory rate of the research group existed less than that of the control group immediately after insertion of the gastroscope, but 1.5 min, 2 min, 2.5 min, 3 min, 5 min, and 7 min after administration, the investigation cluster's respiratory frequency displayed greater compared to the control group, and there are statistically significant differences between groups (*p* < 0.05). The SPO_2_ of the test group displayed greater compared to the control group at baseline and after administration of various time points above. The IPI value of the research group was significantly lower than that of the control immediately after injection, but the 1.5 min, 2 min, 2.5 min, 3 min, and 5 min of the research group displayed considerably larger than those of the control group, and there are statistically significant differences between groups (*p* < 0.05). After 0.5 min, the control's MOAAS score was higher than that of the research group, but the control's MOAAS score was lower than the research group's at 1 min, endoscopy, 2 min, and the end of operation, as shown in Figure 2.

### 3.3. Time-Related Index

The time from the beginning of the administration to the insertion of gastroscope in the research group was about 2.15, 1.97–2.47 min, which was slightly slower than that in the control (1.83, 1.5–2.2 min), and the difference was statistically significant (*p* < 0.05). The awakening time of 8.37 min, was also slightly slower than that of the control group (7.08, 4.65–9.16 min), and the difference was statistically significant (*p* < 0.05). The time from the completion of administration to 4 minutes of IPI and the total examination time was similar between the two groups (*p* > 0.05) as shown in Table 2.

### 3.4. Total Dose of Propofol or RB

In this study, the total dose of remimazolam consumed during operation in the research group was about 0.21 (0.18–0.25) mg/kg, and the sales dose of alfentanil was about 7.27 (7.00–8.33) *μ*g/kg. In the control group, the intraoperative consumption of propofol was about 2.00 (1.00–2.00) mg/kg, and the consumption of alfentanil was about 9.68 (9.09–10) *μ*g/kg.

### 3.5. Intraoperative Adverse Reactions

As shown in Table 3, respiratory depression and hypotension are the most common adverse reactions during operation. The prevalence of hypotension was vastly greater in the investigation group compared with the control group. Furthermore, incidences of cough, body movement, and hiccups in the research group were higher than those in the control group.

### 3.6. Analysis of Doctor and Patient Satisfaction

In this study, the satisfaction of anesthesiologists was 7.83 ± 0.57 in the research group, 7.84 ± 0.48 in the control, whereas the satisfaction of endoscope doctors was 7.89 ± 0.54 in the research group and 7.89 ± 0.47 in the control, respectively.

In addition, the comparison of patient satisfaction is shown in Table 4. In all patients, 34% of the patients in the research test group were very satisfied with the operation, 63% of the patients were satisfied, while 18% of the patients in the control group were very satisfied and 70% of the patients were satisfied. The overall satisfaction rate of the research group was greater than that of the control group, and the difference was statistically significant (*p* < 0.05).

### 3.7. Adverse Reactions within 24 Hours after Operation

As shown in Table 5, the incidence of nausea, dizziness, fatigue, abdominal pain, and abdominal distension in the research group was markedly less than that in the control group.

### 3.8. Regression Analysis

We take the average IPI score as the main measure of the result variables and we adopt the least square method and Probit regression to analyze the results. The two regression results showed that age, sedative, and total dose of analgesia had significant effects on the results, and the covariance coefficient of sedative was 1.57, which indicated that the IPI score of the research group was 1.57 higher than that of the control group.  Table 6 shows the results in detail.

In the meantime, we adopted the XGBoost regression model to predict and analyze the result variables. In Figure 3, we give the importance score of each variable. From the important factor score chart of the IPI average score (Figure 3), we can propose that age has the first influence on IPI score. Furthermore, we analyze the sensitivity of the important variables and analyze the influence of the changes of the important variables on the results when other variables are at their average level. The results of the analysis are shown in Figure 4. Height has no significant effect on blood oxygen content, people with too low height will have low blood oxygen content, and there is no significant difference between ordinary height and tall population. The analgesics will have an impact on satisfaction; groups that need a large number of analgesics will generally not be too satisfied with postoperative satisfaction. In addition, the analgesics will help to improve blood oxygenation. The obvious rule is that the satisfaction of the elderly is higher, and the average IPI score and blood oxygen content (SPO_2_) of the elderly are lower. People with a significant impact on satisfaction, relatively heavy weight are more likely to be satisfied. The average score of IPI will be significantly higher, and the blood oxygen content of overweight people is lower than that of ordinary people.

## 4. Discussion

In clinics, sedative hypnotics and opioid narcotic analgesics are often used in anesthesia induction and maintenance [15]. When two or more drugs are used simultaneously or successively, the drug interaction may occur by modulating the drug action site, competitively binding with the receptor, or affecting the receptor's sensitivity to another drug, that is, synergistic, additive, or antagonistic action [16]. Moreover, synergism and additivity are what we expect, and antagonism is what we want to avoid. The combined use of multiple drugs in intravenous anesthesia, mastering the underlying mechanism of their interaction is very indispensable for the safe and rational use of drugs. In this randomized, single-blind, parallel controlled study, patients undergoing painless gastroscopy were given intravenous anesthesia with alfentanil combined with RB to observe the effects on hypertension, heart rate, oxygen saturation, muscle tremor, injection soreness, and other intraoperative and postoperative adverse reactions and to explore the safety and comfort of alfentanil combined with RB in patients undergoing painless gastroscopy.

Remimazolam is a new type of water-soluble ultra-short-term anesthetic sedative [17]. Previous animal experiments and clinical trials have shown that remimazolam is safe and effective in anesthesia and sedation [9]. Different from the traditional intravenous anesthetics propofol and midazolam, remimazolam is rapidly hydrolyzed by nonspecific plasma esterase in vivo. In the single dose study, it was found that the average dose of remimazolam in 0.01–0.30 mg/kg reached the peak of plasma concentration, the metabolism was rapid, and the average retention time of remimazolam in vivo was only 1 × 7 of that of midazolam [18]. Considering that painless gastroscopy is usually performed in the outpatient clinic with limited equipment and conditions, airway and circulation management is particularly important in the anesthesia in painless gastroscopy. Although the continuous infusion time is more than 2 hours, the maximum half-life is still between 7 and 8 minutes, so it is considered that remimazolam can be administered more accurately than some slow-acting intravenous anesthetics [8]. In addition, different from other benzodiazepines, remimazolam is not easy to cause injection pain because of its water-soluble characteristics, which makes patients more comfortable.

Propofol is the most commonly used intravenous anesthetic to induce and maintain anesthesia, but it cannot be denied that propofol has an inhibitory effect on the cardiovascular and respiratory systems in a time-and dose-dependent manner, which limits its application in grass-roots hospitals with insufficient anesthesiologists and poor resuscitation conditions. The results of this study reveal that all patients can achieve a stable level of sedation in a smooth gastroscopy, but there are great differences in vital signs and operation details between the two groups. Of note, the HR and BP of the patients in the research group and the control group declined to varying degrees. In the implementation of painless gastroscopy, we are most concerned about respiratory inhibition. We are hoping to find a drug regimen that can maintain a moderate depth of anesthesia and, most importantly, ensure that breathing is not affected, which is a very challenging problem [19, 20]. The IPI index is a new tool approved by the FDA to reflect the respiratory state of patients during sedation [21]. It is a comprehensive index based on four physiological parameters: etCO_2_, RR, SPO_2_ and PR. In this experiment, we found that the values of RR, PETCO_2_ and IPI of the test group and the control group decreased to their lowest at 2–3 min, but the decrease of the control group was greater. This means that the two groups have effects on the tidal volume, and rhythm of breathing, but the RB combined with alfentanil group is more able to maintain spontaneous breathing than the propofol combined with alfentanil, and the SPO_2_ is also higher at each time point. Our present study demonstrated that the respiratory inhibition rate of the research group was lower than that of the control, which was necessary to support the notion that the interventions such as mask pressurization and oxygen supply to improve respiration are also less.

Furthermore, the MOAA/S mark of the research group was slightly smaller than that of the control group at 0.5 minutes. At each time point, the MOAAS score of the research group was higher than that of the control, which may not be completely equal to the depth of anesthesia reached by the research group with RB and propofol. The MOAA/S score is a simple evaluation method and the sedation level of patients and the difficulty of being affected are different [22]. In the follow-up research, we expect to find a more accurate way to evaluate the sedation level of the painless gastroscope and to explore the difference in the sedation level between RB and propofol.

Concomitantly, the time from administration to complete the insertion of the gastroscope, and the awakening time in the research group was slightly lower than that in the control group. However, the time from the completion of administration to 4 minutes of IPI and the total examination time of the two groups were similar. After using the same dose of analgesics as the background, compared with propofol, RB has a slightly lower sedation depth and a longer awakening time,, but the total examination time of the two groups remains the same.

As we expected, the most common adverse reactions of the two groups in painless gastroscopy were respiratory depression and hypotension. However, the occurrence of respiratory failure and hypertension was vastly smaller in the study group than in the control category. This is consistent with the research results of recording vital signs at each time point during the operation, but the incidence of cough, movement, and hiccups in the research group was higher than that in the control group. We suspect that the depth of sedation achieved by RB is slightly lower than that of propofol, which is different from the results of previous drug clinical trials [22], which may be due to the inconsistency of the sedation depth evaluation system. Another reason is that the drug regimen is different [23]. In this study, we adopted alfentanil instead of fentanyl and remifentanil as analgesics, which requires further research study. The detection index of this study is affected by many factors, which can only assist other hemodynamic indexes to help compare the hemodynamic effects of different doses of RB on patients. Meanwhile, considering the problem of safe drug use, this study only included the effect of a single dose on the hemodynamics of patients during anesthesia induction and whether other doses of RB were induced under anesthesia without increasing the incidence of adverse events, and the hemodynamics of the patients remained stable.

Moreover, there was no significant difference in the satisfaction of anesthesiologists and endoscopes between the two groups, which indicated that there was no difference in subjective feelings between anesthesiologists and endoscopists in the treatment of drug regimens between the two groups in a single-blind way. The patients' satisfaction with RB was higher after painless gastroscopy, which may be related to less injection pain of RB. In the present study, 24 hours after the operation, the patients' satisfaction was still higher than that in the control. Considering that the adverse reactions such as nausea, dizziness, fatigue, abdominal pain, and abdominal distension in the research group were lower than those in the control, which was due to the fact that RB had little effect on the respiratory and circulatory function of the patient; moreover, postoperative nausea, dizziness, and other adverse reactions are also a new advantage of analgesia. This study still has some shortcomings. First, the quality of this study is limited due to the small sample size we included in the study. Second, this research is a single-center study, and our findings are subject to some degree of bias. Therefore, our results may differ from those of large-scale multicenter studies conducted by other academic institutes. This research is still clinically significant and further in-depth investigations will be carried out in the future.

In conclusions RB and alfentanil have little effect on the respiratory and circulatory function of the patient, in concert with fewer postoperative adverse reactions and higher patient satisfaction, which can provide safe and effective sedation for gastroscopy.

## Figures and Tables

**Figure 1:** General clinical data in the research group and control group.

**Figure 2:** Comparison of vital signs in the research group and control group.

**Figure 3:** The important factor score chart of the IPI average score.

**Figure 4:** The sensitivity of the important variables.

**Table 1:** Patient demographic characteristics.

	Research group	Control group
Patients, *n*	457	457
Male/female	211/246	209/248
Mean age,year(±SD)	52.69 ± 13.12	52.56 ± 12.69
Mean BMI(±SD)	23.97 ± 3.40	23.84 ± 3.50
ASA classification		
I	0	0
II	457	457
Apfel	1.38 ± 0.75	1.40 ± 0.75

**Table 2:** Comparison of time-related indexes between two groups.

Index	Research group	Control group	*p* value
Effective time	2.15 (1.9–2.47)	1.83 (1.5–2.2)	<0.001
The time from completion of administration to when IPI reaches 4 points.	1.52 (0.93–1.73)	1.33 (1.02–1.80)	0.665
Total examination time	8.25 (6.25–10.57)	8.28 (6.48–10.56)	0.624
Awakening time	8.37 (5.74–10.63)	7.08 (4.65–9.16)	<0.001

**Table 3:** Intraoperative adverse reactions.

	Control group (n = 457)	Research group (n = 457)	*p* value
Cough	46 (5.69%)	7 (1.53%)	0.001
Body movement	83 (11.6%)	29 (6.13%)	0.005
Burp	35 (4.6%)	4 (0.66%)	<0.001
Snoring	8 (0.66%)	2 (0.44%)	0.69
Hypotension	70 (14.86%)	50 (6.51%)	<0.001
Respiratory frequency	13.53 (10–17)	13.32 (10–16)	0.32

**Table 4:** A comparison of patient satisfaction between the two groups.

	Very satisfied	Satisfied	Median	Dissatisfied	Very dissatisfied
Research group	151 (34.2%)	279 (63.3%)	9 (2%)	2 (0.5%)	0 (0%)
Control group	84 (18.7%)	312 (69.5%)	50 (11.1%)	3 (0.7%)	0 (0%)

**Table 5:** Adverse reactions within 24 hours of operation.

	Research group (*n* = 451)	Control group (*n* = 456)	*p* value
Feel nausea	44 (5.76%)	71 (14.98%)	<0.001
Vomiting	16 (2.09%)	4 (0.84%)	0.143
Dizzy	51 (6.68%)	32 (6.75%)	1.00
Dizziness	5 (0.65%)	11 (2.32%)	0.024
Headache	9 (1.18%)	5 (1.05%)	1.00
Drowsiness	11 (1.44%)	4 (0.84%)	0.507
Lack of strength	33 (4.32%)	43 (9.07%)	0.001
Stomach swollen	14 (1.83%)	35 (7.38%)	<0.001
Abdominal pain	10 (1.31%)	18 (3.80%)	0.008

**Table 6:** Regression analysis via IPI score.

	*Least square regression*			*Probit regression*		
	Coefficient	*Z* value	*p* value	Coefficient	*Z* value	*p* value
(Int)	6.6774	4.787	0.000	0.4238	1.19	0.2342
Sex	−0.0010	−0.007	0.9942	−0.0002	−0.006	0.9951
Age	−0.0186	−5.285	0.000	−0.0047	−5.26	0.000
Height	−0.0060	−0.679	0.4975	−0.0015	−0.671	0.5023
Weight	0.0061	1.068	0.2859	0.0016	1.059	0.2901
Surgical history	−0.1088	−0.673	0.5013	−0.0278	−0.675	0.4997
Past history	0.0299	0.231	0.817	0.0077	0.234	0.8148
Smoking history	0.2302	1.781	0.0753.	0.0588	1.775	0.0762.
Sedative drugs	0.4159	4.075	0.000	0.1059	4.063	0.000
Total sedative dose	0.0005	1.007	0.3141	0.0001	1.006	0.3146

## Data Availability

The datasets used and analyzed during the current study are available from the corresponding author upon reasonable request.

## Additional Points

*Key Points*. 1. Compared with propofol and alfentanil, RB and alfentanil have little effect on the respiratory and circulatory function of the patient. 2. RB and alfentanil have fewer postoperative adverse reactions and higher patient satisfaction than propofol and alfentanil. 3. RB and alfentanil can deliver secure and efficient sedation.
